# Growth and Development in Preterm Infants and Maternal Parenting Stress after WeChat-Based Extended Care

**DOI:** 10.1155/2022/9987891

**Published:** 2022-06-28

**Authors:** Lan Zheng, Zengxia Zhu

**Affiliations:** ^1^Department of Neonatology, Dongxihu People's Hospital of Wuhan, Wuhan, China; ^2^Operating Room, Dongxihu People's Hospital of Wuhan, Wuhan, China

## Abstract

**Objective:**

WeChat-based extended care has been widely applied in clinical practice such as preoperative assistance in children with congenital heart disease and children with ventricular septal defect. In this study, we aimed to explore the impacts of WeChat-based extended care on the growth and development of preterm infants (PIs) and the nursing satisfaction of their family members.

**Methods:**

From June 2019 to August 2021, 85 PIs and their mothers were selected as the research participants. Among them, 46 pairs receiving WeChat-based extended care were served as the WeChat group, and 39 pairs receiving routine extended care were taken as the control group. After 6 months of intervention, the two groups of PIs were compared in terms of physical development, IQ, and neurological and gastrointestinal functions. For mothers, their psychological states were assessed after intervention using the self-rating anxiety/depression scale (SAS/SDS), and the nursing satisfaction was counted.

**Results:**

After nursing intervention, better physical and IQ development of PIs were observed in the WeChat group compared with the control group (*P* < 0.05). The WeChat group also had notably reduced level of neuron-specific enolase (NSE) and s100*β* protein related to nerve function than that in the control group and exhibited significant higher levels of serum gastrin (GAS) and motilin (MTL) associated with gastrointestinal function (*P* < 0.05). Besides, the WeChat group presented lower SAS and SDS scores and higher nursing satisfaction than the control group in delivery women (*P* < 0.05).

**Conclusion:**

WeChat-based extended care can effectively improve the growth and development and various physical functions of PIs. At the same time, it is helpful to improve maternal psychological states and nursing satisfaction of delivery women, which is worth of clinical application.

## 1. Introduction

Preterm birth is defined as the condition of not reaching a certain gestational period. In healthy women with low-risk pregnancy, there may also be a certain proportion of premature infants. According to the data of the World Health Organization, preterm infants (PIs) refer to those born before 37 weeks of pregnancy or infants less than 259 days from the first day of a woman's last menstruation [1]. Since China has carried forward an overall two-child policy, the number of women with advanced maternal age has gradually increased, resulting in an increasing in the rate of premature delivery [2]. Unlike normal babies, PIs are with shorter gestational age, lighter weight, and undeveloped or immature organs; thus, they are prone to suffer from complicated diseases, which threaten the development of newborns [3]. According to statistics, the global PIs mortality rate has reached 20.8% and is on the rise, posing an important global health issue [4]. Thanks to the continuous development of medical technology, the rescue rate and survival rate of PIs have been significantly improved [5]. However, due to the lack of intrauterine nutrition reserve, PIs have many adverse characteristics and will still face long-term growth and development problems after discharge, causing a heavy burden to their families [6]. Therefore, effective protection of the life and health of PIs and ensurance of their normal development in a sustained and diversified way have become a focus and difficulty in clinical research.

Extended care is a common nursing approach in clinical nursing intervention for PIs. Its core is to continuously provide quality guaranteed treatment services for patients from hospitalization to postdischarge, that is, to extend in-hospital care services and solve the health problems that patients face in life [7, 8]. Therefore, the implementation of extended care for PIs is an important contributor to improve the long-term prognosis of children [9]. With the rapid development and diversified use of the Internet, extended care based on Internet social media has been applied in clinical practice. For instance, WeChat and other communication tools are conducive to rapid communication between doctors and patients by real-time mastering the physical condition and detailed information of patients after discharge [10, 11]. The WeChat-assisted care model was effective in reducing weight gain and preventing gestational diabetes mellitus in overweight pregnant women or pregnant women with obesity [12]. WeChat miniprograms were beneficial to promote mother's own milk feeding of PIs in the neonatal intensive care unit [13]. However, clinical reports on the impacts of WeChat-based extended care on the prognosis, growth, and development of PIs and family care satisfaction are still being explored. This work studies the application of WeChat-based extended care in PIs, providing effective reference and guidance for promoting PIs' prognosis, growth, and development.

## 2. Methods

### 2.1. Study Subjects

From June 2019 to August 2021, 85 pairs of mothers whose pregnancy outcome were premature and their babies were selected as the research participants. Among them, 46 pairs receiving WeChat-based extended care were served as the WeChat group, and 39 pairs receiving routine extended care were taken as the control group. There were 24 infants delivered naturally and 22 infants were delivered by cesarean section in the WeChat group. The control group consisted of 21 women with natural delivery and 18 women with cesarean delivery. The women in the WeChat group were graduated from junior high school and below (9 cases), senior high school and secondary specialized school (15 cases), and junior college and above (22 cases). The control group included 6 women with level of junior high school and below, 12 women with level of senior high school and secondary specialized school, and 21 cases with level of junior college and above. This study has obtained the informed consent of the PIs' families and been approved by Ethics Committee of Dongxihu People's Hospital of Wuhan. Inclusion criteria were as follows: be in accordance with diagnostic criteria of PIs, such as 28 weeks < gestational age <37 weeks and birth weight <2500 g [1]; Apgar score >7 points and PIs with stable condition; single birth; complete clinical data; and mother as the main caregiver has normal communication skills. Exclusion criteria were as follows: congenital diseases; babies who cannot be breastfed; metabolic, hematological, and/or immune diseases; and inability to receive complete treatment for various reasons.

### 2.2. Intervention Protocols

Delivery women and PIs in the control group received routine nursing during hospitalization. Routine maternal and infant examinations were performed, and prevention and treatment of all kinds of diseases of PIs were carried out. In addition, an appropriate temperature of the ward for PIs was ensured, and the incubator was prepared. Infant feeding procedures were strictly followed. The vital signs of PIs were monitored continuously, and respiratory care and daily soothing were carried out. A series of routine extended interventions for discharged PIs were performed, including physical development training (such as head control training, body balance training, and limb muscle strength training) and neuropsychological development healthcare (auditory and visual training for 0-month-old infants, tactile training for 1–3-month-old infants, and 4–6-month-old autonomous awareness practice). Delivery women were trained to master parenting knowledge, (such as breastfeeding, complementary feeding, nutrition calculation, baby sleep intervention, skin management, vaccination, and complication prevention). Nursing methods included discharge guidance, outpatient follow-up, and telephone follow-up.

On the basis of treatments of the control group during hospitalization, WeChat-based extended care was given to the WeChat group after discharge. First, a nursing group including the attending physicians was set up in the department, and a WeChat group was built to carry out WeChat-based extended care with a complete intervention program. Taking time as the stage, the intervention program was divided into 3 stages including 0 months old, 1–3 months old, and 4–6 months old. The intervention content of each stage was defined, and the nurses were responsible for quality control. The main family members including delivery women were trained to master the basic functions of WeChat, such as the reception and release of messages including text, voice picture, and video. After birth, the growth and development needs of PIs were evaluated according to the physical information of infants and their parents, and corresponding nursing plans and breastfeeding programs were worked out. After discharge, PIs' intellectual, physical, and psychological development will be tested, and corresponding trainings were sent to the WeChat group through pictures, video, and words, which was convenient for supervision of nursing situation of each family. Delivery women were instructed to learn the significance and skills of breastfeeding, so as to cultivate the children's sense of security through breastfeeding. In addition, the prevention and treatment of common diseases were informed, so that parents can timely respond to emergencies and reduce risks. The knowledge of scientific child-rearing health education was transmitted through the WeChat group to help parents form a correct concept of child-rearing. What is more, delivery women and their families (especially the spouse) were encouraged to participate in the whole process of continuous nursing intervention for PIs and give feedback of the growth and development of PIs to specialized nurses. After discharge, the medical staff interacted with parents through text, video, and voice via WeChat to eliminate parents' anxiety. The numbers of message readings were checked after sending relative knowledge through the WeChat group each time, and delivery women or family members were informed to reply and participate in online questionnaire. As for the family who failed to view the message and answer the questions twice, the nurses will supervise them by telephone. The PIs were given staged growth and development rehabilitation training, and the combination of family staged development support nursing and regular return visits was implemented, thus enriching the sensory stimulation, language, motor training, cognitive ability and social ability of PIs, and promoting the recovery of their nervous system and motor functions.

### 2.3. Main Outcome Measures

The development of weight, body length, and head circumference of PIs after 6 months of intervention was analyzed. The IQ development in both cohorts of PIs after intervention was evaluated by using the developmental quotient (DQ) scale [14], which includes five evaluation dimensions: adaptation, gross motor, fine motor, language, and social behavior. Lower scores correspond to lower IQ. The alterations of neurological function indexes of PIs, including neuron-specific enolase (NSE) and s100*β* protein, were detected after intervention. The postintervention gastrointestinal function indexes of PIs, including serum gastrin (GAS) and motilin (MTL), were also quantified. The centrifugation was performed to blood sample prior to collection of serum. GAS and MTL were detected by a microplate reader with kits. For the assessment of maternal psychological state after intervention, self-rating anxiety/depression scale (SAS/SDS) [15, 16] was used. Cronbach's alpha for all scales was more than 0.8. The satisfaction evaluation for nursing intervention was also investigated [17].

### 2.4. Statistical Processing

SPSS 23.0 was employed for data processing. A chi-square test was used to compare the count data recorded as percentage between groups. For measurement data represented by (mean ± standard deviation), a *t*-test was used if the data were normally distributed, and a paired *t*-test was adopted for within-group comparisons pre and postintervention. *P* < 0.05 indicates the difference is statistically significant.

## 3. Results

### 3.1. Physical Development of PIs after Receiving WeChat-Based Extended Care

PIs' clinical baseline data including gestational age, gender, birth weight, and ethnic group were compared between the WeChat group and control group. We found that no statistically significant difference was revealed between the two groups (*P* > 0.05, Table 1), suggesting that the two groups are comparable. PIs' weight, body length, and head circumference were considered as outcomes of physical development. The data showed that the weight, body length, and head circumference of PIs in the WeChat group developed better than that in the control group after intervention (*P* < 0.05, Table 2), indicating WeChat-based extended care intervention contributed to better physical development of infants.

### 3.2. IQ Development of PIs after Receiving WeChat-Based Extended Care

PIs' IQ development was assessed using the DQ scale. The results showed that PIs in the WeChat group scored higher on DQ scale than in the control group in adaptability, gross motor, fine motor, language, and social behavior (*P* < 0.05, Table 3). It demonstrated that WeChat-based extended care was beneficial to IQ development of PIs in the WeChat group compared with the control group.

### 3.3. Neurological Function of PIs after Receiving WeChat-Based Extended Care

Similarly, we further evaluated the neurological development of PIs through the detection of nerve injury markers. The test results showed notably lower NSE and s100*β* protein levels in the WeChat group compared with the control group (*P* < 0.05, Table 4), which revealed WeChat-based extended care may decrease the neurological impairment of PIs.

### 3.4. Gastrointestinal Function of PIs after Receiving WeChat-Based Extended Care

Gastrointestinal function is also one of the key indicators for the growth and development of PIs. Thus, GAS and MTL of PIs were measured to evaluate their gastrointestinal function. It was found that the WeChat group had higher GAS and MTL than the control group (*P* < 0.05, Table 5), indicating that the gastrointestinal function of the PIs in the WeChat group is better.

### 3.5. Maternal Parenting Stress after Receiving WeChat-Based Extended Care

The maternal psychological evaluation showed that no difference in SAS and SDS scores was observed between the two groups prior to intervention (*P* > 0.05). However, the postintervention scores of SAS and SDS were notably lower in the WeChat group versus the control group (*P* < 0.05, Table 6), which indicated maternal psychological states in the WeChat group was better. Finally, the results of satisfaction survey showed that the total satisfaction of delivery women in the WeChat group was 95.65%, which was higher than that of 76.92% in the control group (*P* < 0.05, Table 7), indicating that WeChat-based extended care has gained higher recognition.

## 4. Discussion

At present, preterm birth has become a very common risk event in clinical obstetrics and gynecology, with over 20% of pregnant women having premature delivery [18]. For PIs, they face an extremely high possibility of development defects due to insufficient gestation time in the mother's womb [19]. Therefore, it is necessary to provide more professional and targeted postpartum care for PIs in clinical practice, so as to provide them with more reliable safety guarantee. In recent years, most studies have put forward individualized nursing programs for PIs [20, 21], but all of them are limited by the limited hospitalization time of delivery women, resulting in the inability to achieve the implementation of long-term and stable nursing services. While, the extended care intervention is mainly carried out through oral education at discharge and regular follow-up calls after discharge to inquire about relevant information, which lacks attention to patients, causing patients' low self-importance and poor self-management level [22]. Therefore, how to effectively address this shortcoming is of great significance for PIs. WeChat, as the most popular real-time contact APP in China, enables extremely high real-time interaction, which can effectively solve the implementation limitations of extended care at this stage. At this stage, no clinical study has confirmed the influence of WeChat-based extended care on PIs, so this study has important reference significance for future clinical practice.

This study evaluated the influence of extended care based on WeChat through the changes of PIs' body, IQ, and neurological and gastrointestinal functions after nursing intervention. The experimental results showed better conditions of PIs in the WeChat group in all the abovementioned aspects, indicating that extended care based on WeChat can effectively improve the growth and development of PIs. Shen et al. presented a study of WeChat-assisted perioperative care in children with congenital megacolon, indicating WeChat application contributed to improve parents' nursing level, leading to reduce difficulty in defecation and the occurrence of common complications [23]. Gao et al. also demonstrated that, as for the infants undergoing enterostomy, their parents received WeChat-assisted health education and had better nursing ability and less psychological burden, which was helpful to reduce complications of infants, such as mucosal oedema and allergic dermatitis [24]. As we all know, the risk of premature birth is mainly concentrated in the growth retardation and restriction of PIs [25, 26]. Although clinical nursing can provide excellent and professional medical services for PIs, these services cannot be continued after the maternal and children are discharged from the hospital [27]. Therefore, the other nursing focus is to continue to perform accurate and effective nursing work after the short-term in-hospital treatment. Through WeChat, nurses can learn about the situation of children in real time, adjust nursing measures timely, and improve the pertinence of care. At the same time, by means of video education and online questioning, the knowledge about infant care of delivery women and their families can be strengthened, thus enhancing the safety of PIs. In addition, communication and experience sharing among mothers of PIs through the WeChat platform also helps to improve the protection of premature babies more effectively.

Furthermore, lower SAS and SDS scores were determined in the WeChat group in the maternal psychological state survey, indicating that WeChat-based extended care can also effectively improve the psychological state of delivery women. For women, childbirth is a very important stage in their lives, but the ensuing hormone level and role alterations, as well as family member change, are likely to cause violent mood swings in puerperal women. If not dealt with and adjusted in time, it will cause psychological barriers of patients, which is not conducive to their physical and mental health [28]. The occurrence of preterm birth increases the likelihood of maternal anxiety and depression [16]. Traditional nursing methods only work during the period of maternal hospitalization, ignoring home care after discharge [29]. Apart from that, with the continuous improvement of maternal physical condition, their families began to gradually reduce their attention, which made the mother feel an obvious sense of loss [30]. While under the intervention of WeChat-based extended care, pregnant women can not only know more and more professional knowledge of neonatal care but also get enough encouragement and care from the communication with medical staff and other delivery women, so as to quickly find their own ways to relieve anxiety and depression. This not only contributes to the psychological safety of delivery women but also enables the mothers to be more actively involved in the care of PIs, contributing to more ideal results. The survey results of nursing satisfaction also showed a higher over total satisfaction degree in the WeChat group, which confirmed the high application value of extended care based on WeChat.

Of course, we still need to include more research subjects and extend the experimental period to obtain more comprehensive experimental results, such as 20-item neonatal behavioral neurological assessment at the time of discharge and 12 months after discharge. Furthermore, this article failed to present the results of mastery of PIs nursing knowledge in each group. Besides, the strategy and details of WeChat-based extended care need to be constantly improved to provide more accurate and effective care services for premature delivery women and their babies. In conclusion, WeChat-based extended care is worthy of clinical application in terms of improvement in the growth and development of PIs and maternal psychological states along with nursing satisfaction.

## Figures and Tables

**Table 1:** Clinical data of PIs.

Group	*n*	Gestational age (weeks)	Male/female	Birth weight (kg)	Ethnic group Han/ethnic minorities
WeChat group	46	31.3 ± 1.8	25 (54.4)/21 (45.6)	2.2 ± 0.6	45 (97.8)/1 (2.2)
Control group	39	31.0 ± 1.6	22 (56.4)/17 (43.6)	2.4 ± 0.5	36 (92.3)/3 (7.7)
*χ* ^2^/*t*		0.805	0.036	1.651	1.433
*P*		0.423	0.849	0.103	0.231

**Table 2:** Physical development of PIs between two groups after intervention.

Group	*n*	Body mass (kg)	Head circumference (mm)	Height (cm)
WeChat group	46	3.62 ± 0.36	34.68 ± 1.49	49.52 ± 1.73
Control group	39	3.17 ± 0.39	3.2.11 ± 1.39	46.88 ± 1.69
*t*		5.527	8.170	7.085
*P*		<0.0001	<0.0001	<0.0001

**Table 3:** IQ development of PIs between two groups after intervention.

Group	*n*	Adaptability (score)	Gross motor (score)	Fine motor (score)	Language (score)	Social behavior (score)
WeChat group	46	91.65 ± 2.80	91.91 ± 2.67	93.28 ± 1.96	94.39 ± 2.10	91.78 ± 2.60
Control group	39	87.26 ± 2.14	88.28 ± 2.03	86.67 ± 1.59	89.10 ± 1.83	86.49 ± 2.78
*t*		8.005	6.954	16.870	12.270	9.055
*P*		<0.0001	<0.0001	<0.0001	<0.0001	<0.0001

**Table 4:** NSE and s100*β* level related to neurological function of PIs after intervention.

Group	*n*	NSE (ng/mL)	s100*β* (ug/L)
WeChat group	46	14.33 ± 1.93	0.49 ± 0.11
Control group	39	20.21 ± 1.99	1.15 ± 0.19
*t*		13.800	19.960
*P*		<0.0001	<0.0001

**Table 5:** Gastrointestinal function concerning GAS and MTL level in PIs after intervention.

Group	*n*	GAS (ng/L)	MTL (ng/L)
WeChat group	46	391.75 ± 19.29	0.49 ± 0.11
Control group	39	338.11 ± 22.23	1.15 ± 0.19
*t*		11.880	5.514
*P*		<0.0001	<0.0001

GAS, serum gastrin; MTL, motilin.

**Table 6:** Maternal psychological status before and after intervention.

Group	*n*	Before intervention (SAS score)	After intervention (SDS score)	*t*	*P*
WeChat group	46	55.13 ± 4.33	42.72 ± 4.35	14.77	<0.0001
Control group	39	55.23 ± 4.44	49.23 ± 8.53	4.108	0.0002
*t*		0.104	4.531		
*P*		0.9167	<0.0001		

SAS, self-rating anxiety scale; SDS, self-rating depression scale.

**Table 7:** Satisfaction evaluation of nursing intervention.

Group	*n*	Highly satisfactory	Satisfaction	Dissatisfaction	Total satisfaction of delivery women
WeChat group	46	29 (63.04)	15 (32.61)	2 (4.35)	95.65%
Control group	39	11 (28.21)	19 (48.72)	9 (23.08)	76.92%
*χ* ^2^					6.571
*P*					0.010

## Data Availability

The data used to support the findings of this study are included within the article.
